# Ecological strategy of *Phyllostachys heteroclada* oliver in the riparian zone based on ecological stoichiometry

**DOI:** 10.3389/fpls.2022.974124

**Published:** 2022-10-31

**Authors:** Xiong Jing, Wenhui Su, Shaohui Fan, Huiying Luo, Haoyu Chu

**Affiliations:** Key Laboratory of National Forestry and Grassland Administration, International Centre for Bamboo and Rattan, Beijing, China

**Keywords:** riparian zone, *Phyllostachys heteroclada*, aerenchyma, radial oxygen loss, PSII, ecological stoichiometry

## Abstract

The abnormality of seasonal water level fluctuation in the riparian zone causes various ecological and environmental problems, such as vegetation degradation, biodiversity reduction, soil erosion, and landscape transformation, thereby critically modifying the ecosystem structure and functions. This necessitates the development of a dominant vegetation zone with competitive potential. In this study, we investigated the content and distribution pattern of nutrient elements in each organ of the dominant bamboo species, *Phyllostachys heteroclada*, in the riparian zone. We also analyzed the morphological characteristics, root aeration tissue structure, root oxygen exchange capacity, ATP supply situation, and leaf PSII photosynthetic mechanism of two bamboo species (*P. heteroclada* and *P. nigra*) in the riparian zone. Compared with *P. nigra*, the roots of *P. heteroclada* formed well-developed oxygen storage and transport structure, i.e., aeration tissue, and exhibited root oxygen secretion in the waterlogging environment of the riparian zone, whereas the roots maintained a high ATP content through energy metabolism, thus benefiting mineral absorption and transport. Moreover, the accumulation of N, P, Ca, Mg, and Fe in the leaves of *P. heteroclada* was greater under waterlogging conditions than under non-waterlogging conditions, which is the basis for the efficient operation of the photosynthetic mechanism of the leaves. Compared with waterlogged *P. nigra*, the PSII electron acceptor Q_A_ of *P. heteroclada* leaves had a vigorous reducing ability and showed higher efficiency of light uptake energy as well as higher quantum yield indexes ϕ(Eo) and ϕ(Po). This study demonstrates that the ecological adaptive regulation strategies of *P. heteroclada* in the riparian zone are intrinsic driving factors affecting their stoichiometric characteristics, including changes in the absorption and transport of minerals caused by root aeration structure and energy metabolism. Moreover, carbon production and allocation may be caused by the stable photosynthetic mechanism and source-sink relationship of leaves. Through the synergistic regulation of different organs realizing their roles and functions, *P. heteroclada* developed ecological stoichiometry characteristics adapted to the riparian zone.

## Introduction

The riparian zone is a special interlacing area between terrestrial and aquatic ecosystems formed by seasonal water-level fluctuation. The periodic water level fluctuation and human activities cause a series of ecological and environmental problems in the riparian zone, such as vegetation degradation, biodiversity reduction, soil erosion, and landscape deterioration, and in some instances even lead to the loss of a few ecological functions (Décamps et al., 2009; Gumiero et al., 2013; Arif et al., 2021a; Yang et al., 2021).

Maintaining a continuous and competitive (functional) vegetation zone (i.e., ecological adaptation zone) in the riparian zone is necessary for realizing important ecological functions, such as material exchange and energy flow in terrestrial and aquatic ecosystems and water purification (Janssen et al., 2019; Ye et al., 2020; Arif et al., 2021b; Xia et al., 2021). The cloning property of bamboo, especially *Phyllostachys heteroclada*, an important waterlogging-tolerant bamboo species, gives bamboo an obvious advantage when applied to riparian zone restoration and enhances its application prospects when coupled with its once-planted, everlasting use (Cao et al., 2015). Changes in plant nutrient storage and productivity in response to the environment undoubtedly have a vital cascading effect on the variability of biomes and even ecosystem function (Sistla and Schimel, 2012).

As a discipline of the chemical elemental composition of living organisms and the energy balance of ecosystems, phyto stoichiometry has been widely used to study the effects of vegetation on soil ecosystems (Wang et al., 2020a). Studies on the stoichiometry of the riparian zones have focused on soil elements under hydrological changes, such as the relationship between soil chemistry and vegetation community characteristics (Ye et al., 2019) and soil nitrogen metabolism and denitrification (Groh et al., 2020; Zhao et al., 2022). Given the important role of riparian vegetation in the ecological function of the riparian zone, the focus of some studies has shifted to the ecological adaptation characteristics of riparian zone vegetation (Dufour et al., 2019). Adapted plants in the riparian zone can modify their metabolic pathways or adaptive mechanisms to adapt to the waterlogged environment (Rzewuski and Sauter, 2008), such as adjusting their photosynthetic capacity and biomass allocation patterns (Visser et al., 2000; Cho et al., 2021), forming aeration tissues (Qi et al., 2019; Duarte et al., 2021), and forming adventitious roots (Chen et al., 2002; Li et al., 2006; da Costa et al., 2020). These regulations considerably affect plant nutrient uptake and plant growth and development, thereby influencing the characteristics of plant ecological stoichiometry; this provides a theoretical basis for using stoichiometry to link plant organ functions to their ecological adaptation. However, fewer studies have evaluated the ecological adaptation strategies of riparian zone vegetation based on stoichiometry. To overcome these challenges, using ecological stoichiometry as a research link between plant nutrients and growth and its environmental ecological adaptation strategies is important for studies on the ecological restoration of vegetation and soil and water conservation, as well as those relating to the function and succession of the riparian ecosystem (Sterner and Elser, 2002; Tian et al., 2018; Ye and Zhang, 2018; Nóbregaa et al., 2020).

We hypothesized that the ecological adaptation strategy of *P. heteroclada* based on its stoichiometric characteristics has the intrinsic stability of elemental metabolism physiology and the holistic elemental dynamic balance; that is, the allocation of the minerals and photosynthetic products (total C) to overground and underground organs is a trade-off in favor of ecological adaptation in the riparian zone, which is supported by the stable root energy metabolism and photosynthetic mechanism. We thus proposed three study objectives: to investigate the cumulative distribution and interactions of minerals based on root oxygen uptake and energy metabolism; to elucidate the accumulation and distribution of carbon based on the function of photosynthetic organs in leaves; and to analyze the ecological adaptation strategies of *P. heteroclada* in combination with the stoichiometric characteristics of its important nutrients. This study established a new perspective on the ecological adaptation strategies of adapted plants in the riparian zone; our findings may serve as a reference for other studies assessing vegetation in the ecological environment of the riparian zone of other river basins based on the stoichiometry characteristics and the application of *P. heteroclada* to the riparian zone restoration.

## Materials and methods

### Study area and plant materials

Taiping Lake area (Figure 1), the research site, is located in the upper reaches of the Qingyi River, west of Huangshan City, southern Anhui Province, with a total area of more than 86 km^2^. Taiping Lake is a deep-water artificial alpine lake that has merged with various streams and rivers flowing into the upper reaches of the Qingyi River, adjacent to Jiuhua Mountain in the north and Huangshan Mountain in the south. It is known as Lake Geneva in the east. This area is part of the subtropical monsoon climate zone, with an annual sunshine duration of ca. 1,647.6 h, an annual average temperature of ca. 15°C, an annual average frost-free period of 235 days, annual precipitation of ca. 800–1,600 mm, and more rainfall in June and less in December (Hu, 2018). Taiping Lake, as an artificial detention reservoir with an annual pondage of 2.4 billion m^3^, can impound 1/3 of water flow in the flood season, ensuring downstream farmland production and residents' safety along the river. Even as the Taiping Lake riparian zone plays the ecological function of the land-water interlacing area, it is important to understand the ecological adaptability of its own vegetation.

**Figure 1:** Taiping Lake location and the detail of the riparian zone.

The plants in the riparian zone of the Taiping Lake basin are mainly herbaceous plants, such as annual *Poaceae, Asteraceae*, and *Leguminosae*, specifically *Phragmites australis, Alternanthera philoxeroides, Bidens frondosa, Paspalum paspaloides*, and *Erigeron annuus* (Hu, 2018). Some tree species, such as *Metasequoia glyptostroboides* and *Pinus massoniana*, are also scattered. Bamboo has outstanding ecological value as a clonal plant in the riparian zone, with its rapid forest establishment and high ornamental value. In view of the vegetation investigation of the Taiping Lake riparian zone (Cao et al., 2015; Hu, 2018), this study used the waterlogging-tolerant type of dominant bamboo species (*P. heteroclada*) in Taiping Lake as the test material.

### Experimental setup

The experiment was a factorial design with two bamboo varieties and two water conditions [normal water treated (CK) and waterlogging stress (WS)]. One-year-old clones of *P. heteroclada* were used as test materials growing in the riparian zone of Taiping Lake, and 1-year-old *P. nigra* (same genus and similar diameter and height) was used as control.

The test materials were planted in pots (45 cm diameter, 30 cm high, one seedling per pot) with ~15 kg of soil from the riparian zone. For the WS group, the pots were placed in a pool that was dug previously at a depth of ca. 40 cm and infused with water to ensure that all the roots of the seedlings were submerged. The seedlings in the CK group were watered normally, ensuring that water did not accumulate at the bottom of the pots. Twenty replicate pots were conducted for each treatment.

### Measurement of mineral elements and C content

On days 3, 6, 9, 12, and 15, fresh leaves, branches, stems, and fine roots were sampled from *P. heteroclada* after WS or CK treatment. Three replicate plants were randomly sampled for each treatment at each time point. There were measured by destructive plant sampling. The samples were processed in two steps: green removal at 105°C for 30 min and drying at 65°C to constant weight. The dry samples were ground and sieved to determine the mineral and carbon (C) content. Total C was determined using the potassium dichromate (K_2_Cr_2_O_7_) oxidation-heating method. Total nitrogen (N) was determined using the semi-micro Kjeldahl method, with the sample digested by sulphuric acid-hydrogen peroxide (H_2_SO_4_-H_2_O_2_). Total phosphorus (P) was determined using the molybdenum antimony antispectrophotometric method, with the sample digested by H_2_SO_4_-H_2_O_2_. Calcium (Ca), iron (Fe), and magnesium (Mg) content were determined using inductively coupled plasma mass spectrometry (ICP-MS; Teledyne Leeman Labs, Hudson, NH, USA).

### Analysis of aerenchyma histological images and air cavity area calculation using laser confocal microscopy luminescence

The fresh roots of *P. heteroclada* and *P. nigra* were sampled after 15 days of waterlogging stress treatment. The maturation zone of the roots was subjected to a HitoCore NANOCUT R-automatic rotary microtome (Leica, Berlin, Germany) for sectioning. The image of the root tissues was observed through lignin autofluorescence excited by an excitation wavelength of 498 nm by using a confocal laser microscope (LSM 880 NLO, Zeiss, Oberkochen, Germany). In addition, the root imaging data of *P. heteroclada* and *P. nigra* under CK and WS treatments were imported into ZEISS ZEN Lite (blue edition) software for the histological observation and calculation of the aerenchyma in the air cavity area of the roots (sample root air cavity area = total area of section air cavity/total area of section surface).

### Oxygen flux rate in roots detected using non-invasive micro-test technology

After waterlogging stress treatment for 15 days, the O_2_ flux in the root tips of *P. heteroclada* and *P. nigra* was measured using non-invasive micro-test technology (NMT) (NMT Physiolyzer, Younger USA LLC, Amherst, MA 01002, USA, Xuyue Company, Beijing, China), as described by Yuan et al. (2021), with some modifications. In brief, the root samples were rinsed with distilled water, fixed at the bottom of the petri dish, and then stood in the test solution (0.1 mmol CaCl_2_, 0.1 mmol KCl, pH 6.0) for 30 min. Next, the test solution was discarded, and 5 mL of fresh test solution was added for sample testing. Points on the root surface ~5,000 μm from the tip of the root tip were selected to observe O_2_ fluxes. At least three samples were measured for each treatment.

### Measurement of ATP content

Root samples from seedlings of the WS and CK treatments were collected and snap-frozen. For each treatment, 1 mL of solution for sample extraction was added into the mortar by using a pipette (Finnpipette, Finland) to be ground with ~0.1 g root tissue. The solution was then transferred to a centrifuge tube, homogenized in an ice bath, and centrifuged at 12,000 rpm at 4°C for 10 min using a micro high-speed centrifuge (TG16W, Hunan, China). The supernatant was sampled and placed on ice in preparation for testing. The samples were spotted on an ELISA kit and detected using an enzyme marker (Rayto, RT-6100, Jinan, Shandong, China).

### Imaging of stem vascular tissue

A confocal laser microscope (LSM 880 NLO, Zeiss, Oberkochen, Germany) was used to scan the vascular tissues in the transverse section of the stem of *P. heteroclada* at 498 nm, while the vessels and sieve tubes of the vascular bundle were scanned and analyzed separately using a Hitachi S-4800 scanning electron microscope (Hitachi High-Technologies Corporation, Tokyo, Japan).

### Measurement of chlorophyll fluorescence rise kinetics

The healthy leaves on the branch in the upper-middle zone of *P. heteroclada* and *P. nigra* were used to measure chlorophyll fluorescence rise kinetics at room temperature with a Handy-PEA fluorometer (Plant Efficiency Analyzer, Hansatech Instruments Ltd., King's Lynn, Norfolk, UK), as described by Chen et al. (2016). After 20 min, the light probe was docked to the dark-adapted clip, and then the lightproof sheet metal was opened to examine the OJIP polyphasic chlorophyll (Chl), fluorescence rise kinetics, and JIP-test of *P. heteroclada* and *P. nigra* by continuous excitation fluorometer (Handy PEA, Hansaech, UK). The difference in the physiological status of photosynthesis between *P. heteroclada* and *P. nigra* under WS and CK treatments was analyzed, including the PSII reaction process, photochemical activity, light energy absorption, and conversion efficiency.

### Statistical analysis

Data were analyzed using Excel 2019 (version 16.64) (Microsoft, Redmond, Washington, USA), SPSS (version 19.0) (SPSS Inc., Chicago, IL, USA), and RStudio software (version 3.6.2) (R Core Team, 2020) products. All experiments were conducted at least three times. The values were expressed as the mean ± standard error (SE) of the mean. Data were subjected to analysis of variance through the Tukey (HSD) test or Student's *t*-test to determine significant differences. A significant difference was considered at *P* < 0.05. FactoMineR and other program packages in RStudio were used for principal component analysis, and eigenvectors and eigenvalues, and cumulative contribution rates of the sample correlation matrix were calculated.

## Results and discussion

### Accumulation and allocation of minerals of *P. heteroclada* based on root oxygen uptake and energy metabolism

#### *P. heteroclada* shows efficient mineral uptake and allocation in the riparian zone

The effective absorption and allocation of minerals in plant tissues are important for riparian zne-tolerant species to survive under waterlogging stress. Roots are known as the main organs of plants to absorb minerals. Nutrient elements are mainly transported and allocated by the xylem or phloem, which is believed to be closely related to the nutrient requirements of plant organs. Meanwhile, minerals in the riparian zone water body have a large impact on the local aquatic ecosystem as follows: eutrophication caused by overmuch N and P in the water body, water quality, hardness influenced by Ca and Mg content, water turning yellow, and water pollution caused by excess Fe content, and so on (Xu et al., 2005). Therefore, effective mineral uptake and accumulation by adaptive plant roots in the riparian zone provides the material basis for plant metabolism, which plays a restorative role in the aquatic ecosystem in riparian zones. We evaluated the accumulation and allocation of nutrients (N, P, Mg, Ca, and Fe) among different tissues, namely leaves, branches, stems, and roots of *P. heteroclada* after waterlogging in the riparian zone. Waterlogging conditions triggered a holistic alteration in the nutrient allocation of *P. heteroclada*. With the extension of the test time, from 9 to 15 days, waterlogging treatment promoted the accumulation of N in the leaves and branches of *P. heteroclada* but obviously decreased N content in the stems and roots (Figure 2A). Meanwhile, the P content increased significantly in the leaves from 6 to 15 days but decreased in the roots almost the whole time after the waterlogging treatment (Figure 2B). We suggest that the decrease of N and P content in *P. heteroclada* roots resulted from waterlogging in the riparian zone, and N and P were mainly allocated to the leaves to support the healthy operation of the photosynthetic apparatus, which lays a foundation for chlorophyll formation and efficient photosynthetic electron transfer in plants. These allocation patterns of important minerals affect the biostoichiometry of *P. heteroclada* (Agren et al., 2012; Kobayashi and Tanoi, 2015). In addition, the accumulation of Ca^2+^, a critical second messenger in plant abiotic stress resistance (Lee and Seo, 2021), in both leaves and roots was promoted by waterlogging treatment at 15 days. Calcium content decreased in stems and branches from 3 to 15 days, while the Ca content in leaves initially decreased (3 days) and then increased from 9 to 15 days, but Ca content in the roots initially decreased from 3 to 9 days and then increased from 12 to 15 days after waterlogging treatment (Figure 2C), which may be related to the resistance physiology of *P. heteroclada* roots and leaves under waterlogging. The trend of Mg content was similar to that of Ca content (Figure 2D). We also observed a significantly higher Fe content in the roots of waterlogging-treated plants from day 6 to day 15 than in the control plants (Figure 2E). Notably, the formation of Fe plaques in the roots, which is closely associated with aerenchyma development and O_2_ state, can improve the nutritional status of plants (Mei et al., 2014). Meanwhile, an increased accumulation of Fe was observed in *P. heteroclada* leaves after the waterlogging treatment. The strong ability of the *P. heteroclada* root to absorb Fe provides a reference for the application of *P. heteroclada* for ecological restoration in iron-polluted aquatic environments.

**Figure 2:** Effects of waterlogging treatment on the accumulation pattern of N **(A)**, P **(B)**, Ca **(C)**, Mg **(D)**, and Fe **(E)** in the leaf, branch, stem, and root of *Phyllostachys heteroclada*. Data and bars represent the means ± SE of three independent replicates. Asterisks indicate the significant differences between treatments (*P < 0.05, **P < 0.01, ***P < 0.001, *t-test*). WS, Riparian zone waterlogging stress.

Typically, N, P, Ca, Mg, and Fe accumulation increased in the leaves, while N and P content decreased in the roots of *P. heteroclada* after the waterlogging treatment (Figure 2). In summary, we can conclude that the waterlogging treatment mainly affects the reallocation rather than the nutrient accumulation of these minerals in *P. heteroclada* organs. These results suggest the reallocation of the absorbed minerals among the organs might be a nutrient-associated physiological strategy for *P. heteroclada* in response to waterlogging. These factors affect the interaction between the elements. Moreover, *P. heteroclada* in the riparian zone had lower N and P concentrations in its stems, branches, and roots than in its leaves, irrespective of whether it is in a waterlogged environment. This may be related to the dilutive effect of water on nutrients, since the stems, branches, and roots have to store and provide substantial quantities of water and nutrients for leaves to maintain the stability of their own photosynthetic production.

#### Adaptive strategies for oxygen uptake and energy metabolism in the roots of *P. heteroclada* in the riparian zone

The biggest problem faced by the plants in the riparian zone is a reduction in the oxygen (O_2_) supply caused by the slow diffusion rate and limited solubility of O_2_ in water, which results from waterlogging (Limami et al., 2014). Reduction in energy (ATP) production negatively triggered by oxygen deficiency induces a significant decline in minerals (ion) absorption and transport (Visser et al., 2003; Colmer and Greenway, 2011; Loreti et al., 2016; Li et al., 2017; Shen et al., 2020). For instance, waterlogging reduces K, Ca, and Mg accumulation in wheat plants (Sharma et al., 2018). Noticeably, the adaptive plants in the riparian zone can show different coping strategies based on genetic diversity under the O_2_-deficient condition caused by waterlogged stress, including morphological and metabolism adaptations. Some of the above strategies are adventitious root formation, stem elongation growth, and aerenchyma tissue formation to ensure the O_2_ supply and energy generation (Bailey-Serres and Voesenek, 2008; Jin et al., 2013; Narsai and Whelan, 2013; Fukao et al., 2019).

The increased formation of aerenchyma represents a morphological adaptive strategy for plants suffering from hypoxic stress (Colmer, 2003; Hossain and Uddin, 2011). Aerenchyma is a continuous oxygen transport channel that provides a low-resistance internal pathway for the movement of O_2_ from the aerobic shoots to anaerobic roots to facilitate plant aerobic respiration under hypoxia or oxygen-poor conditions (Justin and Armstrong, 1987; He et al., 1996; Gunawardena et al., 2001; Duarte et al., 2021; Evans and Carvalho-Evans, 2021; Sou et al., 2021). We examined the aerenchyma of *P. heteroclada* adapted to waterlogged stress in the riparian zone, with *P. nigra* as a control. The results showed that the aerenchyma increased in the root tissues of both *P. heteroclada* and *P. nigra*. However, *P. heteroclada* showed stronger aerenchyma formation under waterlogging conditions (Figure 3A). Moreover, a significant interaction between the bamboo species and the water conditions was observed; the waterlogging-induced increase in aerenchyma (calculated under waterlogging/normal conditions) was more obvious in the waterlogging-tolerant *P. heteroclada* (13.04-fold) than in the waterlogging-sensitive *P. nigra* (4.74-fold) (Figure 3B).

**Figure 3:** Effects of waterlogging treatment on the formation of aerenchyma **(A,B)**, O_2_ flux **(C)**, and ATP production **(D)** in the roots of *Phyllostachys heteroclada* and *P. nigra*. Data and bars represent the means ± SE of at least three independent replicates. Asterisks indicate the significant differences between treatments (*P < 0.05, **P < 0.01, ***P < 0.001, *t-test*). WS, waterlogging stress.

The increase in aerenchyma formation provides a low-resistance oxygen transport channel for root cell metabolism, reducing the number of oxygen-consuming cells in the roots; it also discharges part of the exhaust gas out of the body and allows part of the oxygen to be transported to the roots to penetrate the surrounding soil, forming a small oxygenated rhizosphere to create an aerobic environment for inter-root microorganisms and effectively impedes the accumulation of toxic components (Hayashi et al., 2013; Watanabe et al., 2013; Armstrong and Armstrong, 2014; Evans and Carvalho-Evans, 2021; Sou et al., 2021). Waterlogging-tolerant plants respond to waterlogging stress by developing barriers that impede radial O_2_ loss into the rhizosphere. Some waterlogging-tolerant plant species can form an apoplastic barrier deposited by suberin or lignin on the outer cell layers of roots to reduce radial oxygen loss (ROL) from the aerenchyma and prevent toxic compounds from entering the root, For example, some wheat genotypes can increase suberin or lignin on epidermis or exodermis of the root, which may act as barriers against ROL and result in increased tolerance to waterlogging (McDonald et al., 2001; Sauter, 2013; Watanabe et al., 2013). This is because the formation of aerenchyma and barriers increases internal aeration efficiency, providing a pathway for O_2_ diffusion from shoots to submerged roots. We discovered a significant interaction between the bamboo species and the water conditions in which the net flux rate dynamics of O_2_ shifted from influx to outflux in the roots of waterlogged-tolerant *P. heteroclada*, while the O_2_ influx had a significant decrease (waterlogging vs. control, ca. 4.3 fold) in the roots of waterlogging-sensitive *P. nigra* (Figure 3C). This finding indicates that the O_2_ provided to the roots of *P. heteroclada* is probably absorbed by the strong tissue spaces of aerenchyma. Notably, the ROL of *P. heteroclada* was discovered at 20,000 μm from the root tip under waterlogging, while the same part of *P. nigra* roots nearly cannot absorb O_2_ from the soil. The O_2_ flux close to 0 femtomole·cm^−2^·s^−1^, which may be related to the less formation of *P. nigra* adventitious root after waterlogging and more severe root rot and lignification in the roots due to harmful substances produced by anaerobic respiration. These contrasting results thus indicate an oxygen metabolism-dependent strategy in waterlogging-tolerant species under hypoxia stress. Oxygen is crucial for ATP generation to drive mineral element ion transport. Hypoxia stress caused by waterlogging can provoke mitochondrial dysfunction and impair energy metabolism (Wagner et al., 2018). However, ATP production in the roots was not compromised in waterlogged *P. heteroclada*, whereas ATP production in *P. nigra* roots was significantly inhibited by waterlogging, which might be due to the mitochondrial respiration of *P. heteroclada* enhanced by an increased O_2_ supply (Figure 3D).

In summary, *P. heteroclada* showed stronger aeration tissues to provide oxygen to the roots and higher ATP content than *P. nigra* in the waterlogged environment (Figure 3). We suggest that these adaptive strategies guarantee the efficient operation of mineral element absorption and distribution in the roots of *P. heteroclada*. Notably, the pattern of mineral element uptake and allocation of the roots of *P. heteroclada* was more beneficial and inclined to the leaves in the riparian zone (Figure 2), (wherein N and Mg as elements of chlorophyll, P involved in the transformation of intermediate products and energy transfer of photosynthesis, and Fe played the role of electron transfer in leaf photosynthetic metabolism), as minerals absorbed by the roots could collectively guarantee the robust operation of photosynthetic mechanisms in the leaves in the waterlogged environment. The above conclusion was verified by evaluating the phenotypic response of *P. heteroclada* and *P. nigra* to waterlogging conditions, while normal morphological characteristics are tied to the stable operation of the physiological mechanism. At 6 and 15 days post-waterlogging treatment, *P. nigra* leaf growth was strongly inhibited, as deemed from the wilting, yellowing, and withering leaves, as common symptoms for plants under waterlogging conditions; by contrast, *P. heteroclada* growth was not compromised, as gleaned from lack of visible damage. This indicates that *P. heteroclada* leaves were healthier than *P. nigra* leaves under waterlogging stress (Figure 4).

**Figure 4:** Morphological comparison of *Phyllostachys heteroclada* and *P. nigra* in the riparian zone. Bars, 16 cm. WS, waterlogging stress.

The adaptation of *P. heteroclada* to the riparian zone is expressed not only in the above-ground leaf morphology but also in the changes in root morphological characteristics, such as the number of new roots, the length of fine roots, root rot, and lignification. *P. nigra* had a reduced number of adventitious root formations and more serious root rot and lignification in waterlogging conditions (Figure 4 and Table 1). Poor root aeration is generally considered the main cause of root rot and lignification, which may be related to toxic substances produced by the roots of *P. nigra* in oxygen-poor conditions.

**Table 1:** Effects of waterlogging treatment on the root characteristics of *Phyllostachys heteroclada* and *P. nigra* under waterlogging conditions.

**Bamboo species**	**Treatment**	**The number of adventitious roots**			**The fresh weight of adventitious root (g)**
		**0–1 cm**	**1–5 cm**	**5–10 cm**	
*P. heteroclada*	Control	183.33 ± 19.60a	95.00 ± 13.64a	17.66 ± 2.49a	3.77 ± 1.15a
	WS	178.00 ± 19.62a	64.33 ± 4.99b	15.00 ± 1.63a	3.37 ± 0.81ab
*P. nigra*	Control	158.33 ± 13.89ab	83.00 ± 5.72ab	14.33 ± 1.89a	3.10 ± 0.67ab
	WS	112.67 ± 7.59b	18.00 ± 4.55c	5.33 ± 1.24b	1.10 ± 0.16b

Dates represent the means ± SE of three independent replicates. Different letters indicate significant differences between the treatments (analysis of variance with Duncan's test, P < 0.05).

In addition, plants adapt to heterogeneous soil conditions by altering their hydrophytic root architecture; for example, lateral roots can branch through hydro patterning when the roots are in contact with water (Maurel and Nacry, 2020). Water availability is a potent regulator of plant development and induces roots to branch through hydro patterning (Eysholdt-Derzsó and Sauter, 2017; Orosa-Puente et al., 2018; Robbins and Dinneny, 2018). Plants under waterlogging probably replace the original root system with adventitious roots by activating a mechanism (Sauter, 2013). We measured the adventitious root formation of both *P. heteroclada* and *P. nigra* under waterlogging. Table 1 presents the numbers of adventitious roots (1–10 cm) of *P. nigra* that were significantly decreased by the waterlogging treatment. However, in waterlogging-tolerant genotypes *P. heteroclada*, the number of adventitious roots decreased only by 1–5 cm, but that of the others at 0–1 and 5–10 cm was maintained high. Some studies have concluded that short roots are usually “windows” for radial O_2_ loss instead of an adaptive mechanism. Notably, the formation of adventitious roots (0–1 cm) of *P. heteroclada* did not significantly change the quantity under waterlogging treatment. Our data showed that the 0–1 cm adventitious roots of *P. heteroclada* have few aerenchymas, thus limiting the loss of oxygen. Notably, our study found that the number of long roots (5–10 cm) had no significant change in *P. heteroclada* under waterlogging, whereas that of *P. nigra* decreased significantly. Hayashi et al. (2013) found that maintaining root length density can be one of the essential traits for waterlogging tolerance to maintain shoot growth. This is related to sustaining water uptake and the resulting photosynthesis under waterlogged conditions.

In addition, the fresh weight of adventitious roots of *P. nigra* decreased, whereas that of *P. heteroclada* was not affected by waterlogging conditions, probably due to the internal accumulation of metabolic carbohydrates. Consistently, waterlogging caused smaller damage (displayed as fold change of root number and fresh weight under waterlogging stress) on *P. heteroclada* than *P. nigra*, demonstrating that an adventitious root system might be necessary for *P. heteroclada* to tolerate waterlogging stress in the riparian zone.

In conclusion, *P. heteroclada* can adapt to waterlogging stress in the riparian zone by changing the absorption and allocation pattern of minerals, including N, P, Ca, Mg, and Fe, between the above and below ground parts of the plant. Efficient oxygen transport of aeration tissues, uncompromised cellular energy metabolism, and morphological adaptations of roots may be key factors in rational absorption and a trade-off allocation of minerals.

### Carbon accumulation and distribution pattern of *P. heteroclada* based on the leaf photo response system

#### Total carbon source-sink transport and characteristics of distribution and accumulation in various organs of *P. heteroclada*

Photosynthesis is an important production mechanism for organic matter in plants, converting carbon dioxide and water into organic matter through light reactions (e.g., photosynthetic electron transfer) and carbon assimilation. Plant total C content reflects its organic matter content, and total C plays a vital role in driving plant stoichiometry, such as C:N and C:P changes, which are also linked with the cycling processes of elements such as N, P, and S (Lal, 2004).

The vascular system provides objective conditions for transporting photosynthetic products from the source leaf to sink organs of *P. heteroclada*. Because lignin deposition is crucial for vascular system formation, we used a laser confocal microscope to study the structure of the vascular bundle of *P. heteroclada* stem by lignin autofluorescence, taking advantage of the high lignin content in the vascular bundle. The results show that the vascular system of the *P. heteroclada* stem contains multiple vascular bundles, each of which consists of two vessel elements (VE) and a sieve tube (ST) with sieve holes. We observed that the vascular bundles were arranged in a V-shaped scattering pattern on the transverse section by observing the transection structure of *P. heteroclada* stems. At the bottom of the V-shape was an ST, and the arms of the V-shape each had two VE (Figure 5A). The vascular system provides pathways for the transportation of allocated photosynthetic products produced by the leaves of *P. heteroclada* and is also essential for the redistribution of water and minerals absorbed by the roots in the organs. Minerals such as N, P, Mg, and Fe are transported to the leaves through the VEs to maintain a stable continuation of photosynthetic mechanisms (Figure 2). Waterlogging stress probably inhibits photosynthetic products from being transported from leaves to roots, leading to the accumulation of carbohydrates in plant leaves (Topa and Cheeseman, 1992). Waterlogging stress also imposes restrictions on the underwater gas exchange of the roots, resulting in energy and carbohydrate deficits in the roots (Sasidharan and Voesenek, 2015; Cho et al., 2021). However, our research showed that the accumulation of total C content due to outward transport inhibited by waterlogging did not occur in *P. heteroclada* leaves in the riparian zone, and no significant decrease was noted in the total C content of the roots except on days 3 and 12 (Figure 5B). *P. heteroclada* might be capable of allocating more C to the root through the vascular system, thereby increasing the root C reservation. The ability of plants to adapt to waterlogging stress is related to maintaining the energy supply to the underground part of cell life activities (Peña-Fronteras et al., 2009). This hypothesis is also verified by our results that the ATP content of the roots of *P. heteroclada* was not significantly decreased in the waterlogged environment of the riparian zone, and the well-developed aeration tissues of the roots guarantee oxygen supply for cellular respiration in the roots of *P. heteroclada* (Figure 3).

**Figure 5:** *Phyllostachys heteroclada* stem structure images. Vascular bundles are marked as (VB), sieve tubes are marked as (ST), and vessel elements are marked as (VE) **(A)**; Effects of waterlogging treatment on the allocation pattern of total C in *P. heteroclada* **(B)**. Asterisks indicate the significant differences between treatments (*P < 0.05, ***P < 0.001, t-test).

The source-sink relationship model suggests that allocating assimilation results from the interaction of all sources, sinks, and transport pathways (Daudet et al., 2002). When the supply of assimilates is limited, the priority of sinks determines the order in which they acquire assimilates. Assimilates are allocated to satisfy the demand of sinks with higher priority first, followed by allocation to organs with a lower priority if a surplus exists. Photosynthetic products are transported through the phloem, and transport capacity is determined using the source-sink unit, which is formed in relation to the growth pattern of each organ, the direction of the vascular bundle, and the distance between organs. The Munch pressure flow theory stipulates that the transport flux of assimilates in the vascular bundle is driven by the turgor pressure gradient, which can be illuminated using the flux calculation formula (J = δP·C·k, where δP is the gradient of turgor between source and sink, C is the concentration of assimilates, and k is equal to the conductivity coefficient) of the assimilates in the vascular bundle (Satchivi et al., 2000). The formula for the conductivity coefficient of the phloem is k= A.r2/8η.l (where A is the cross-sectional area of the phloem; r is the radius, and η is the viscosity coefficient; l is the length of the phloem from source to sink; r does not vary much in the plant organs).

In summary, *P. heteroclada* produces photosynthetic products through CO_2_ assimilation of photosynthesis in source leaves and allocates photosynthetic products produced by source leaves to plant organs in the form of carbon for storage by STs. The transport intensity of photosynthetic products from source to sink is determined using the photosynthetic rate, the cross-sectional area of the primary phloem, the length between source and sink, and the concentration of assimilates. The carbon allocation pattern between *P. heteroclada* organs shows ecological adaptation characteristics to the environment of the riparian zone. In addition, the ability of plants to adapt to waterlogging in the riparian zone cannot be estimated merely by the carbohydrate content before and after waterlogging or by the efficiency of carbohydrate utilization by plants (Das et al., 2005).

#### Efficient photosynthetic electron transport is typical of *P. heteroclada* to respond to riparian zone waterlogging conditions

Photosynthesis is a basic physicochemical process for plant growth and survival and is greatly affected by water conditions (Gao et al., 2018; Yan et al., 2018; Dalal, 2021). Waterlogging affects carbon assimilation in plants (Pezeshki, 2001; Pedersen et al., 2013; Garcia et al., 2020). For instance, waterlogging stress results in decreased carbohydrate content and biomass accumulation in *Arundinella anomala* and *Salix variegate* (Ye and Zeng, 2013). However, healthy and efficient light-responsive photosynthetic electron transfer is necessary for photosynthetic carbon assimilation in *P. heteroclada*. We evaluated the physiological conditions of the photosystem electron transfer chain of *P. heteroclada* after different waterlogging treatments, using *P. nigra* as a control.

The OJIP curve was used to verify the level of PSII electron transfer in *P. heteroclada* and *P. nigra* leaves. As the PSII reaction center of the leaf is partially closed, the fluorescence will increase in the O-J phase, and the increase in the J point indicates the reduction of electron transfer efficiency from Q_A_ to Q_B_ in the PSII reaction. This study showed differences in the O–J phase between *P. heteroclada* and *P. nigra* at different stages under different waterlogging stresses. Specifically, the value of the J point of waterlogging-treated *P. heteroclada* was lower or equal to that of control plants. The value of J point was significantly increased in *P. nigra* after waterlogging treatment for 10 h and 20 h, which is hypothesized to be evidence of ${\text{Q}}_{\text{A}}^{-}$accumulation due to slowed outward electron transfer of Q_A_ (Figure 6A). It was found that the electron transfer efficiency from Q_A_ to Q_B_ of both *P. heteroclada* and *P. nigra* increased during the initial stage (<5 h) of waterlogging stress compared with CK. However, the electron transfer efficiency from Q_A_ to Q_B_ of *P. nigra* decreased significantly after waterlogging treatment for 10 h. Similarly, waterlogging conditions caused vulnerability to photosynthesis and PSI of the waterlogging-sensitive *Helianthus tuberosus* L (Yan et al., 2018). However, waterlogging-treated *P. heteroclada* showed non-compromised electron transfer efficiency in the late stage of waterlogging compared with the control plants. Significantly, *P. heteroclada* exhibited a strong reducing ability of Q_A_, PSII electron acceptor, under waterlogging conditions, which was related to the physiological state of the leaf photosynthetic apparatus. This is likely because *P. heteroclada* roots guaranteed the efficient absorption of essential minerals required by the leaf photosynthetic apparatus and transported minerals upwards through the vascular bundle for utilization by the leaf photosynthetic apparatus. The I–P phase reflects the PSI-driven electron flow from PQH_2_ to the end electron acceptors on the PSI acceptor side. After waterlogging treatment, both *P. heteroclada* and *P. nigra* showed a trend of rising and then decreasing fluorescence IP-amplitude (ΔF_IP_). Notably, the ΔF_IP_ and ΔV_IP_ of the *P. heteroclada* were higher than those of *P. nigra* in different stages of the waterlogging treatment. When Q_B_ accepts electrons from ${\text{Q}}_{\text{A}}^{-}$ and forms ${\text{Q}}_{\text{B}}^{2-}$, Q_A_ and Pheo completely enter the reduced state, and the PSII reaction center is completely closed and no longer accepts light quanta. The fluorescence yield is the highest by this time, leading to the appearance of the P point (Chen et al., 2016). The above results revealed that waterlogging-treated *P. heteroclada* had stronger photosynthesis than waterlogging-treated *P. nigra* (Figure 6B).

**Figure 6:** Effects of waterlogging treatment on the photosynthetic efficiency of *Phyllostachys heteroclada* and *P. nigra* under waterlogging conditions. Comparative analysis of the typical Chl fluorescence induction kinetics OJIP **(A)**, “O” marking the original point of fluorescence and “P” marking the fluorescence peak; fluorescence IP-amplitude ΔF_IP_ and ΔV_IP_, Different letters indicate significant differences between treatments (analysis of variance with Duncan's test, *P* <0.05) **(B)**; analysis of variance contribution rate of all principal component of JIP-test parameters **(C)**; the principal component analysis (PCA) of JIP-test parameters **(D)**; a radar plot presentation of some important JIP-test parameters quantifying the behavior of PSII, all values are expressed compared with the values of control **(E)**. The experiment was performed with at least three replicates.

Next, we analyzed the kinetic parameters of fluorescence of *P. heteroclada* and *P. nigra* using principal component analysis (PCA). The results revealed that the variance contribution rates of the first three principal components were 54.7, 16.9, and 11.9%, respectively; the matrix eigenvalues were 4.9593, 2.7539, and 2.3184, which could represent 83.5% of the comprehensive information of the physiological characteristics of the fluorescence parameters evaluated with the JIP test (Figure 6C). The factor loading contribution and correlation analysis showed that the first three principal components represent the state of the leaf photosynthetic apparatus, including the activity of the PSII reaction center and the absorption, conversion, and dissipation of light energy by the photosynthetic organs. The main factors of the JIP test with a high contribution rate were area and the quantum yield of electron transfer ϕ(Eo); the performance indexes were PI Inst., PI abs, and PI total (Figure 6D). Furthermore, the radar chart, drawn by the main factors of the JIP test of *P. heteroclada* and *P. nigra* in response to waterlogging stress screened by PCA, showed that the waterlogging treatment did not significantly affect the maximum photochemical efficiency ϕ(Po) of both *P. heteroclada* and *P. nigra*. However, at the initial stage, PI abs and PI Inst of *P. heteroclada* were higher than those of *P. nigra*, but after waterlogging stress, they were similar between the two plants. Compared with *P. nigra, P. heteroclada* demonstrated a stronger ability to capture, absorb, and transmit light energy per unit area, as well as higher efficiency of absorbed light energy into the electron transport chain and higher maximum quantum yield indicators [ϕ(Eo) and ϕ(Po)] (Figure 6E).

Overall, these results suggest that *P. heteroclada* maintained high photosynthesis compared with the repressed photosynthetic activity of *P. nigra* after waterlogging stress. The healthy functioning of the photosynthetic apparatus of *P. heteroclada* leaves in the riparian zone is inevitably dependent on enough photosynthesis-related minerals provided to photosynthetic organs, which benefit from the rational absorption of nutrients by roots with a good oxygen supply and ATP metabolism. Meanwhile, *P. heteroclada* also adapts to the riparian zone environment by the efficient electron transfer of PSII, the basis for photosynthate supply, and the rational allocation of photosynthate through the source-sink relationship of vascular tissues.

### Ecological stoichiometry characteristics of *P. heteroclada* in the riparian zone and its relationship to ecological adaptation

Nutrient content in organs such as roots, stems, and leaves of plants depends on the dynamic balance between soil nutrient supply and vegetation elemental demand; therefore, ratios of stoichiometry often tend to be stable. For instance, the leaf N:P ratio averages between 11.0 and 15.8 (Reich and Oleksyn, 2004; Han et al., 2005; Tian et al., 2018). Moreover, plant ecological stoichiometry, an important link between plant nutrient uptake and plant growth, is related to the ecological adaptation strategies of different organs of *P. heteroclada* based on their own functions.

Notably, plants' C:N:P stoichiometry has been widely used to infer nutrient limitations and responses to environmental change (Cao et al., 2020; Wang et al., 2020b). We observed that the C:N ratio of waterlogging-treated *P. heteroclada* increased in the roots and stems but decreased in the branch and leaf, and the C:P ratio increased in the branches, stems, and roots, while it decreased in the leaf (Figure 7). The N:P ratio, which showed variability in different organs of *P. heteroclada* in the riparian zone, was higher in leaves under WS than that of CK, had greater variability in the branches under waterlogging, and displayed an increasing trend in the branch with an extension of the waterlogging time, while the stem N:P ratio under WS was lower than that of CK. These results indicated a changed C:N:P stoichiometry of *P. heteroclada* under waterlogging conditions. This study shows that the intrinsic drivers of these changes in stoichiometry characteristics are the combined effects of carbon changes dominated by leaf photosynthesis and mineral absorption characteristics related to oxygen supply and energy metabolism in roots, which are closely interlinked by the vascular system as a pathway for nutrient distribution and transport among organs. Taken together, this constitutes a regulation strategy for each organ of *P. heteroclada*, based on stoichiometry characteristics.

**Figure 7:** Analysis of stoichiometry characterization of C, N, and P elements of *P. heteroclada* in the riparian zone.

Plant C:N and C:P changes depend mainly on leaf nitrogen (N) and phosphorus (P) content, which are important components of the basic structure of plant cells and play a crucial role in the production and transformation of proteins and nucleic acids (Garten, 1976). The absolute content of both and their stoichiometric relationship largely determine the functional properties of photosynthetic processes, plant growth, and reproduction. In our study, higher C:N and C:P ratios were observed in the roots of waterlogging-treated *P. heteroclada* (Figure 7), which was related to the significant reduction of N and P content in its roots (Figure 2). Meanwhile, waterlogged *P. heteroclada* distributed more N and P to the leaves to complete cell proliferation in the riparian zone, causing a decrease in leaf C:N and C:P (Figure 7). The mutual coupling of carbon (C) and nitrogen (N) makes C:N an important indicator for exploring plant element allocation and adaptation strategies. Plants with high C:N have high nitrogen use efficiency and can maintain high C:N in a highly N-limited environment to improve nutrient use efficiency and thus prioritize plant survival, while plants maintaining low C:N in a relatively less N-limited environment are more conducive to competing for resources to achieve rapid growth, and litter with low C:N has the quality of rapid decomposition (Zhang et al., 2020). Notably, this study found that the root C:N ratio of *P. heteroclada* in the riparian zone environment ranged from 28 to 36, and increased with a longer duration of waterlogging, which had a positive effect on the efficient use of nitrogen in waterlogged *P. heteroclada* in the riparian zone and could affect the growth of fine roots.

N:P is a sensitivity coefficient for nutrient limitation of plant growth, and N and P content and balance further affect plant growth characteristics, functional attributes, vegetation productivity (Chapin et al., 1986; Tang et al., 2018), maintenance of community species diversity (Fujita et al., 2010), soil-plant nutrient cycling (Deng et al., 2017), and ecosystem succession (Bobbink et al., 2010). The N:P ratios of *P. heteroclada* leaves were higher in the waterlogging environment than in the non-waterlogging (CK) environment and were relatively stable as the duration of flooding increased. However, the N:P ratios of *P. heteroclada* branches were more variable under waterlogging in the riparian zone, which is consistent with the field experiment on plant N:P reported by Schreeg et al. (2014). Studies on the herb *Eranthis hymalis* have observed that the higher the leaf N:P ratio, the lower the annual growth rate of the plant (Niklas and Cobb, 2005). In addition, experiments based on the model plant (*Arabidopsis thaliana*) also confirmed that the stoichiometry relationship between nitrogen and phosphorus in the reproductive organs of plants is more stable than in other organs to ensure the reproduction of plants (Yan et al., 2016). This study found that the stoichiometry relationship between nitrogen and phosphorus was more stable in leaves and roots than in branches and stems in the riparian zone, which may be related to the synergistic nutrient allocation between different organs adapting to the waterlogging environment in the riparian zone.

Some studies have attempted to define the type of plant nutrient limitation in terms of the N:P ratio. Koerselman and Meuleman (1996) conducted fertilization experiments on wetland vegetation and demonstrated that plant growth was N-limited when the plant's N:P <14 but was regulated by both N and P when N:P was between 14 and 16; in other words, plant growth was not a clear N:P limitation, while plant growth was limited by P when N:P > 16. Güsewell (2004) analyzed all terrestrial ecosystems and revealed that herbaceous plants were N-limited at N:P <15 but P-limited at N:P > 15. Later, some researchers proposed N:P <10 or N:P > 20 as criteria for determining plant growth limited by N or P, respectively. In conclusion, ecological stoichiometry criteria also differ between different ecosystems and different species, making it non-sensical to use a uniform standard to estimate which nutrients limit the ecosystem. In the current study, we observed that the N:P of *P. heteroclada* ranges from 12 to 16 in different water conditions in the riparian zone, whether under waterlogging or not (Figure 7).

These results support the notion that variables (here, waterlogging) in the riparian zone can affect nutrient concentrations and ecological stoichiometry of organs by changing the allocations of C, N, and P among the plant organs. The different environments in which the organs are located and the different roles and functions that the organs play in the plant result in differential characteristics of changes in the stoichiometry of *P. heteroclada* organs in the riparian zone. The internal driving force of this difference is the efficient energy metabolism in the root and the oxygen channel formed by aerenchyma, which jointly supports the absorption of minerals. In addition, the effective production function of photosynthetic apparatus in leaves and the balance and allocation of photosynthetic products (total C) among organs (Figure 8) in *P. heteroclada* exhibits adaptive growth in the environment of the riparian zone through the synergistic ecological stoichiometry characteristics of different organs.

**Figure 8:** Relationship between ecological stoichiometry characteristics and ecological adaptation strategies of *Phyllostachys heteroclada* in the riparian zone.

## Conclusions

In this study, we evaluated the accumulation and distribution patterns of nutrients and stoichiometric characteristics in different organs of *P. heteroclada*, as well as adaptive strategies affecting root mineral uptake and the photosynthetic apparatus relating to the production function of leaf photosynthesis. The following conclusions were obtained:

- The well-developed aeration tissues and stable energy metabolism of the roots of *P. heteroclada* in the riparian zone provide the basis for the uptake, transport, and distribution of minerals, including N, P, Ca, Mg, and Fe. Moreover, the stable photosynthetic mechanism and source-sink relationship of the leaves guarantee the production of photosynthetic organic matter and the allocation of total C. The nutrients distributed to the organs through the vascular system show a trade-off. The above together form the stoichiometric characteristics of different organs of *P. heteroclada* in the riparian zone.
- The ecological adaptation strategies of *P. heteroclada* to the environment of the riparian zone can lead to changes in the accumulation of nutrient configurations in its organs, which also affect its ecological stoichiometry. *P. heteroclada* can adapt to riparian zone waterlogging stress by oxygen reserves provided by well-developed aeration tissues in the roots, ATP content maintained by stable energy metabolism, and efficient operation of photosystems such as healthy PSII in the leaves. These ecological adaptation strategies are intrinsic driving factors of the stoichiometric characteristics of *P. heteroclada* in the riparian zone.
- The vascular system provides a pathway for the distribution and transport of photosynthetic products produced by *P. heteroclada* leaves, and the condition for the redistribution/reconfiguration of water and minerals absorbed by the roots to each organ. *P. heteroclada* are more inclined to transport minerals, including N, P, Ca, Mg, and Fe, to the leaves to guarantee the photosynthetic mechanism to ensure the operation of photosynthesis in the leaves. The photosynthetic products are distributed to the organs according to the source-sink relationship to ensure the healthy growth of *P. heteroclada* in the waterlogging environment of the riparian zone.

## Data availability statement

The original contributions presented in the study are included in the article/supplementary material, further inquiries can be directed to the corresponding authors.

## Author contributions

XJ, WS, and SF conceived the ideas. XJ collected the data, analyzed the data, and led the writing. XJ, HC, and HL proofed the effectivity and rationality of the method proposed in this manuscript. All authors contributed critically to the ideas and drafts and gave final approval for publication.

## Funding

This study was supported by Fundamental Research Funds of ICBR, grant number 1632022019.

## Conflict of interest

The authors declare that the research was conducted in the absence of any commercial or financial relationships that could be construed as a potential conflict of interest.

## Publisher's note

All claims expressed in this article are solely those of the authors and do not necessarily represent those of their affiliated organizations, or those of the publisher, the editors and the reviewers. Any product that may be evaluated in this article, or claim that may be made by its manufacturer, is not guaranteed or endorsed by the publisher.
